RETRACTED

# MiR-486-3p inhibits the proliferation, migration and invasion of retinoblastoma cells by targeting ECM1

**DOI:** 10.1042/BSR20200392

**Published:** 2020-06-04

**Authors:** Hongwei Yang, Yonggang Huang, Jian He, Guangrui Chai, Yu Di, Aiyuan Wang, Dongmei Gui

**Affiliations:** 1 Department of Ophthalmology, Shengjing Hospital of China Medical University, Shenyang, Liaoning, China; 2 School of Mechanical Engineering and Automation, Northeastern University, Shenyang, Liaoning, China; 3 Department of Ophthalmology, Jinzhou Central Hospital, Jinzhou, Liaoning, China

**Keywords:** ECM1, Migration, miR-486-3p, Proliferation, Retinoblastoma

## Abstract

It has been reported that miR-486-3p expression is decreased in retinoblastoma (RB) tumor tissues, however, its function in RB has been less reported. The present study aimed to explore the regulatory effects of miR-486-3p on RB cells. The expression of miR-486-3p in RB tissues and cells was detected by quantitative real-time polymerase chain reaction (qRT-PCR). Cell viability, proliferation, apoptosis, migration and invasion ability were determined by cell counting kit-8 (CCK-8) kit, clone formation assay, flow cytometry, scratch assay and transwell, respectively. Targetscan 7.2 and dual-luciferase reporter were used to verify target genes for miR-486-3p. The expressions of apoptosis-related proteins and ECM1 were detected by Western blot. The miR-486-3p expression was decreased in RB tissues and cells. In RB cells, overexpression of miR-486-3p inhibited cell proliferation, migration and invasion, while promoted apoptosis. Moreover, overexpression of miR-486-3p decreased Bcl-2 expression, while increased the expressions of Bax and Cleaved Caspase-3 (C caspase-3). ECM1 was the target gene of miR-486-3p, and miR-486-3p inhibited the expression of ECM1. Furthermore, ECM1 partially reversed the inhibitory effect of miR-486-3p on the proliferation, migration and invasion of RB cells. MiR-486-3p inhibited the proliferation, migration and invasion of RB by down-regulating ECM1.

## Introduction

Retinoblastoma (RB) is a common intraocular tumor in infants and young children, which seriously endangers the vision and life of children [1,2]. Early and timely treatment of RB patients can achieve better survival rate and retention of visual function [3,4], while the tumor will grow and spread rapidly within the eyeball, invade the vitreous body and subretinal space, spread to the skull along the optic nerve, leading to the death of the patient, without timely diagnosis or treatment [5–7]. At present, the common treatment methods for RB are transpupillary thermal therapy, cryotherapy, chemotherapy, and ophthalmectomy, orbital exenteration and gene therapy [8,9]. Gene therapy is the treatment of a disease by manipulating a therapeutic gene or disease-related gene as a therapeutic target, which has a good prospect in the application of multiple tumor therapies [10,11]. Thus, it is important to explore the biological and molecular mechanisms of RB in order to identify new diagnostic criteria and therapeutic targets.

RETRACTED

MicroRNAs (miRNAs) are non-coding single-stranded RNAs that inhibit or degrade the mRNA by binging with the target mRNA 3′-untranslation region (3′-UTR), and regulate the target genes expression [12–14]. Previous studies have demonstrated that miRNA expression may be specific to certain types of cancer and tumor-derived miRNAs may be stably detected in the plasma or serum [15,16]. In recent years, it has been reported that plasma miR-320, miR-let-7e and miR-21 acted as novel potential biomarkers for the detection of RB [17]. In addition, studies have found that many miRNAs are abnormally expressed in RB, such as miR-192, miR-34a and miR-376a [18–21]. miR-125b promoted tumor growth and suppressed apoptosis by targeting DRAM2 in RB [22]. miR-188-5p promoted epithelial–mesenchymal transition via targeting DNA binding 4 through Wnt/β–catenin signaling in RB [23]. These studies indicate that abnormal miRNA expressed may have some influence on the development of RB. Therefore, the discovery of abnormally expressed miRNAs and their target genes in RB may provide a new idea for the research and treatment of the molecular mechanism of RB.

Studies have shown that miR-486-3p is abnormally expressed in a variety of cancer cells, such as oral cancer, cervical cancer and oral tongue squamous cell carcinoma [24–26]. The down-regulation of miR-486-3p is considered as one of the causes for metastasis of cervical cancer [25]. Venkatesan et al. [27] found that miR-486-3p expression was decreased in the RB tumor tissues, however, the role of miR-486-3p in RB is unclear. In the present study, clone formation assay, flow cytometry, transwell chamber and other experimental methods were used to investigate the effect of overexpression of miR-486-3p on the proliferation, apoptosis and invasion ability of RB, in order to provide new ideas for clinical treatment of RB.

## Materials and methods

### Reagents

RPMI-1640 medium (31870082; Gibco, U.S.A.); 10% fetal bovine serum (FBS, 16140071; Gibco, U.S.A.); 100 U/ml penicillin (10378016; Gibco, U.S.A.); 100 μg/ml streptomycin (10378016; Gibco, U.S.A.); Lipofectamine 2000 Transfection Reagent (11668030; Invitrogen, U.S.A.); Wright’s–Giemsa’s staining solution (G5225; GBCBIO technologies Inc., China); paraformaldehyde (P0099-500ml; Beyotime, China); Crystal Violet (C0121; Beyotime, China); TRIzol reagent (15596026; Invitrogen, U.S.A.); SYBR miRNA detection assays (Takara, China); RIPA buffer (P0013K; Beyotime, China); PVDF membrane (Merck, Germany); Cell counting kit-8 (CCK-8, C0037; Beyotime, China); Annexin V-FITC Apoptosis Detection kit (APOAF; Sigma–Aldrich, U.S.A.); PrimeScript RT Master Mix kit (RR036A; Takara, China); BCA protein assay kit (23225; Pierce, Germany).

RETRACTED

### Clinical samples and cell culture

Human tissue samples (including RB tumor tissues and normal retinal tissues) of 45 patients with RB who were underwent eye enucleation in Shengjing Hospital of China Medical University were collected. All patients were not treated with radiotherapy or chemotherapy before operation, the postoperative pathological sections were diagnosed as RB. The samples were frozen and stored in liquid nitrogen, the tissues used for pathological examination were fixed by 4% paraformaldehyde. The experimental procedure was approved by Ethics Committee of Shengjing Hospital of China Medical University, and the written informed consent of each patient was obtained.

Human retinal pigment epithelial cells (ARPE-19) and RB cell lines (Y79, SO-RB50, WERI-Rb-1) were both purchased from the Typical Cell Culture Collection Committee of the Chinese Academy of Sciences Library (http://www.cellbank.org.cn/search.asp?a=1). All cells were cultured in RPMI-1640 medium containing 10% FBS, 100 U/ml penicillin, 100 μg/ml streptomycin at 37°C with 5% CO_2_.

### Transfection

Transfection of miRNA: Y79 and SO-RB50 were transfected with miR-486-3p mimic (mimic group) or miR-486-3p mimic control (mimic control group) by Lipofectamine 2000 Transfection Reagent, according to the manufacturer’s instructions. The single cell suspension at a density of 5 × 10^4^ cells/ml was prepared and seeded into the 96-well plate. The miRNA was mixed with OPTIM-MEM 1, and then the Lipofectamine 2000 reagent and OPTIM-MEM 1 were added and incubated for 20 min. Then, the mixture was incubated at 37°C with 5% CO_2_ for 48 h. The untreated cells were set up as control group (blank group).

#### Transfection of vector

The expression vector with wild-type/mutant ECM1-3′-UTR sequences was designed and synthesized by Shanghai GenePharma Co., Ltd (China). Y79 and SO-RB50 were co-transfected with miR-486-3p mimic and ECM1-WT or ECM1-MUT. The untreated cells were set up as control group (blank group). The experiment was divided into four groups: blank-ECM1-WT group, mimic-ECM1-WT group, blank-ECM1-MUT group and mimic-ECM1-MUT group. For another transfection experiments, Y79 and SO-RB50 were co-transfected with miR-486-3p mimic control or miR-486-3p mimic and ECM1-WT (ECM1) or empty vector (negative control, NC). The experiment was divided into four groups: Mimic control+NC group, Mimic control+ECM1 group, Mimic+NC group, and Mimic+ECM1 group. The full list of the primers used for transfection are shown in Table 1.

RETRACTED

**Table 1:** The primers for transfection

Name	5′–3′
miR-486-3p mimic	CGGGGCAGCUCAGUACAGGAU
miR-486-3p mimic control	UCACAACCUCCUAGAAAGAUAGA
ECM1	Sense: CAAGATCTATGGGGACCACAGCCAGAGC
	Antisense: CAGGTACCGTTCTTCCTTGGGCTCAGAG
ECM1 negative control	AATTCACTCCAAGTCTCTTCC

### Cell viability assay

CCK-8 kit was performed to determine the cell viability of Y79 and SO-RB50. The cell density was adjusted to 5 × 10^5^ cells/ml and inoculated in a 96-well plate and cultured for 24, 48, 72 h, then the CCK-8 solution was added and again cultured for 2 h. Optical density (OD) of each well was measured at the wavelength of 450 nm by a microplate (Model 680, Bio-Rad, U.S.A.).

### Clone formation assay

Cells were re-suspended in RPMI-1640 and seeded into a 35-mm culture dish with 500 cells per plate, and cultured at 37°C in a 5% CO_2_ cell culture incubator. After 14 days, the cells were fixed with 4% poly-methanol for 20 min, then stained with Wright’s–Giemsa’s staining solution for 10 min. After natural air drying, the images were observed and counted under the inverted phase contrast microscope (CK40, Olympus, Japan).

### Cell apoptosis

The Annexin V-FITC Apoptosis Detection kit was performed to determine cell apoptosis. Cells at the density of 1 × 10^6^ cells/ml were resuspended in binding buffer. Then, the mixture was mixed with Annexin V-FITC and incubated in dark environment for 10 min. The propidium iodide (PI) was added, and then incubated in dark environment for 15 min. Cell apoptosis was analyzed by flow cytometry (BD FACSCalibur, BD Biosciences, U.S.A.).

### Scratch assay

Cells were seeded into a 24-well plate at a density of 5 × 10^5^ cells/ml, and a straight wound was created by a sterile pipette tip. At 0 and 48 h after the wounding, the cells were imaged by inverted phase-contrast microscope (Eclipse TS100, Nikon, Japan) and the cell migration was analyzed by NIS-Element Basic Research v3.2 software (Nikon, Japan).

### Transwell

Transwell chambers (8-μm pores, Corning Company, U.S.A.) pre-coated with Matrigel were placed into a 24-well plate, and the cells were seeded on the upper champers at a density of 2 × 10^5^ cells/well. The serum-free medium was added to the upper chamber, the RPMI-1640 medium with 10% FBS was added to the lower chamber. After 48 h, the excess culture fluid was removed and the invaded cells were fixed with 4% paraformaldehyde for 5 min, and then stained with 0.1% Crystal Violet for 5 min. The image was observed under an inverted microscope (TS100, Nikon, Japan).

RETRACTED

### miRNA target prediction and dual-luciferase reporter assay

The TargetScan 7.2 (http://www.targetscan.org/) was used to predict the potential target of miR-486-3p. The miR-486-3p mimic and ECM1-WT or ECM1-MUT were co-transfected into Y79 and SO-RB50 by Lipofectamine 2000 Transfection Reagent, respectively. The untreated cells were set up as control group (blank group). The luciferase activities were measured using the Dual-luciferase Reporter Assay kit (Promega, U.S.A.).

### Quantitative real-time polymerase chain reaction

Total RNA was isolated from cells by TRIzol reagent. RNA purity and concentration were determined by NanoDrop 2000 (Thermo Fisher Scientific, U.S.A.). The total RNA (2 μg) was reverse transcribed to cDNA by PrimeScript RT Master Mix kit. Then, SYBR miRNA detection assays and Opticon real-time PCR Detection System (ABI 7500, Life Technology, U.S.A.) were used for quantitative analysis. The response procedure: 94°C for 5 min, (94°C for 30 s, 58°C for 30 s, 72°C for 30 s) ×35 cycles, and 72°C for 5 min. The expression level was calculated using 2^−ΔΔ*C*_T_^ method. *U6* was used as internal reference gene, and the primers for quantitative real-time polymerase chain reaction (qRT-PCR) used in the present study were shown in Table 2.

**Table 2:** The primers for qRT-PCR

Name	Forward: 5′–3′	Reverse: 5′–3′
miR-486-3p	GGCAGCTCAGTACAGGATAAA	CGGGGCAGCUCAGUACAGGAU
U6	CTCGCTTCGGCAGCACA	AACGCTTCACGAATTTGCGT

### Western blot

Total protein was lysed with RIPA buffer and then was quantified with BCA protein assay kit. The protein (20 μg) was separated by 10% SDS/PAGE, and transferred to PVDF membrane. The membrane was blocked with 5% skim milk solution for 1 h, and then incubated with primary antibodies overnight at 4°C: anti-Bcl-2 (ab59348, 1:1000, Acbam), anti-Bax (ab32503, 1:1000, Acbam), anti-Cleaved Caspase-3 (C caspase-3, #9661, 1:1000, CST), anti-GAPDH (ab8245, 1:2000, Acbam), anti-extracellular matrix protein 1 (ECM1, ab126629, 1:1000, Acbam). Next, the membrane was incubated with horseradish peroxidase (HRP)–conjugated secondary antibodies for 2 h: goat anti-rabbit IgG H&L (HRP) (ab205718, 1:2000, Abcam), goat anti-mouse IgG H&L (HRP) (ab205719, 1:2000, Abcam). GAPDH was used as a control. The protein band was analyzed by Pierce Western Blotting ECL substrate kit (Thermo Fisher Scientific, U.S.A.) and BandScan 5.0 system (Bio-Rad, Hercules, U.S.A.).

### Statistical analysis

Experiments were repeated at least three times. SPSS 20.0 system (SPSS Inc., U.S.A.) was used for statistical analysis. All experimental data was presented as the mean ± standard deviation (SD). Comparisons between groups were analyzed with Student’s *t* tests or one-way ANOVA. *P*<0.05 was considered to be statistically significant.

RETRACTED

## Results

### miR-486-3p was down-regulated in RB tissues and cell lines

The expression of miR-486-3p in tissues and cell lines (ARPE-19, Y79, SO-RB50, WERI-Rb-1) was measured by qRT-PCR. The miR-486-3p level was lower in RB tumor tissues (RB group) than that in normal retinal tissues (normal group, Figure 1A, *P*<0.05). Moreover, compared with ARPE-19, the miR-486-3p level was lowly expressed in Y79, SO-RB50 and WERI-Rb-1 (Figure 1B, *P*<0.05). Compared with normal tissues and cells, the expression of miR-486-3p was significantly decreased in RB tissues and cells, which may indicate that miR-486-3p was involved in the occurrence and development of RB.

**Figure 1:** The miR-486-3p level in normal and RB tissues and cells were observed (**A**) The human tissue samples were taken from 45 patients with RB who were underwent eye enucleation, qRT-PCR was used to detect miR-486-3p expressions in normal retinal tissues (normal group) and RB tumor tissues (RB group). (**B**) The miR-486-3p expression in ARPE-19, Y79, SO-RB50 and WERI-Rb-1 cell lines were detected by qRT-PCR. (A) **P<0.01 vs. normal; (B) **P<0.01 vs. ARPE-19.

### miR-486-3p was up-regulated by miR-486-3p mimic

Our previous experiments showed that miR-486-3p level was lower in Y79 and SO-RB50; therefore, Y79 and SO-RB50 were selected to investigate the effect of miR-486-3p on RB. Y79 and SO-RB50 were transfected with miR-486-3p mimic control (mimic control group) and miR-486-3p mimic (mimic group), respectively, and a blank group was set. The transfection of overexpressed miR-486-3p was detected by qRT-PCR, and miR-486-3p level was highly expressed in mimic group (including Y79 and SO-RB50) (Figure 2A, *P*<0.05), miR-486-3p mimic up-regulated miR-486-3p expression.

**Figure 2:** The effects of miR-486-3p on cell proliferation and apoptosis were observed (**A**) Y79 and SO-RB50 were transfected with miR-486-3p mimic (mimic group) or mimic control (mimic control group), and a blank group was established, the miR-486-3p expression was detected by qRT-PCR. (**B**) Cell viability of Y79 cells was determined by CCK-8. (**C**) Cell viability of SO-RB50 cells was determined by CCK-8. (**D**) Cloning ability of Y79 and SO-RB50 cells was determined by clone formation assay. (**E**) The clones of RB cells were inhibited by miR-486-3p mimic. (**F**) Apoptosis rates of RB cells were promoted by miR-486-3p mimic. (**G**) Apoptosis of Y79 and SO-RB50 cells was determined by flow cytometry. **P<0.01 vs. Blank, ^##^*P*<0.01 vs. mimic control.

RETRACTED

### miR-486-3p mimic inhibited cell proliferation

Cell viability and the ability of cell cloning were detected by CCK-8 and clone formation assay. As shown in Figure 2B,C, in Y79 and SO-RB50 cell lines, the cell viability was lower in mimic group than that in blank group and mimic control group (*P*<0.05). Clone formation assay demonstrated that the clones in Y79-mimic and SO-RB50-mimic groups were lower than those in corresponding blank and mimic control groups (Figure 2D,E, *P*<0.05). The cell viability and the ability of cell cloning were inhibited by miR-486-3p.

### miR-486-3p mimic promoted apoptosis

For the apoptosis of Y79 and SO-RB50, the apoptosis rate and the expressions of related apoptotic proteins were detected by flow cytometry and Western blot. In Y79 cell line, the apoptosis rate was higher in mimic group than that in blank and mimic control groups (Figure 2F,G, *P*<0.05). Moreover, compared with blank and mimic control groups, in mimic group, Bcl-2 expression was down-regulated, while the Bax and C caspase-3 expressions were up-regulated (Figure 3A,B, *P*<0.05). In addition, in SO-RB50 cell line, compared with blank and mimic control groups, the apoptosis rate (Figure 2F,G) and the Bax and C caspase-3 expressions (Figure 3C,D) in mimic group were up-regulated, and the Bcl-2 expression (Figure 3C,D) was down-regulated (*P*<0.05). We found that miR-486-3p mimic promoted apoptosis.

**Figure 3:** Expressions of Bcl-2, Bax and C caspase-3 in RB cells were observed (**A**) Expressions of Bcl-2, Bax and C caspase-3 in Y79 cells were detected by Western blot. (**B**) In Y79, miR-486-3p mimic decreased Bcl-2 level, and increased Bax and C caspase-3 levels. (**C**) Expressions of Bcl-2, Bax and C caspase-3 in SO-RB50 cells were detected by Western blot. (**D**) In SO-RB50, miR-486-3p mimic decreased Bcl-2 level, and increased Bax and C caspase-3 levels. **P<0.01 vs. Blank, ^##^*P*<0.01 vs. mimic control.

### miR-486-3p mimic inhibited cell migration and invasion

The cell migration and invasion were detected by scratch and transwell. In Y79 and SO-RB50 cell lines, compared with blank and mimic control groups, the cell migration (Figure 4A,B) and invasion (Figure 4C,D) in mimic group were down-regulated (*P*<0.05), suggesting that miR-486-3p inhibited cell migration and invasion.

**Figure 4:** The effects of miR-486-3p on migration and invasion of RB cells were observed (**A**) Cell migration of Y79 and SO-RB50 was determined by scratch assay. (**B**) In Y79 and SO-RB50, cell migration was inhibited by miR-486-3p mimic. (**C**) In Y79 and SO-RB50, cell invasion was inhibited by miR-486-3p mimic. (**D**) Cell invasion of Y79 and SO-RB50 was determined by transwell. **P<0.01 vs. Blank, ^##^*P*<0.01 vs. mimic control.

RETRACTED

### ECM1 was a target gene of miR-486-3p in RB cells

To study the mechanism of miR-486-3p in RB cells, the Targetscan7.2 was performed to predict the target gene and the potential binding sites of miR-486-3p. As shown in Figure 5A, the 3′-UTR of ECM1 contained an area that matched to the miR-486-3p sequence. Then, Y79 and SO-RB50 were co-transfected with miR-486-3p mimic and ECM1-WT or ECM1-MUT to confirm whether miR-486-3p can bind to ECM1, and the dual-luciferase reporter was used to determine the luciferase activity. In Y79 and SO-RB50 cell lines, it was found that the luciferase activity in mimic-ECM1-WT group was reduced, while no reduction was observed in that of mimic-ECM1-MUT group (Figure 5B,C, *P*<0.05), ECM1 was a target gene of miR-486-3p.

**Figure 5:** The potential target of miR-486-3p was predicted and verified (**A**) Targetscan7.2 predicted that ECM1 was a potential target gene of miR-486-3p. (**B-C**) Y79 and SO-RB50 were co-transfected with miR-486-3p mimic and ECM1-WT or ECM1-MUT, and the luciferase activities were measured by dual-luciferase reporter. **P<0.01 vs. Blank.

### miR-486-3p inhibited ECM1 expression

In the present study, the ECM1 vectors (containing 3′-UTR) were transfected into miR-486-3p-expressing RB cells, and a control group was set up. The experimental design was divided into four groups: mimic control+NC group, mimic control+ECM1 group, mimic+NC group and mimic+ECM1 group, and Western blot was performed to confirm ECM1 expression in RB cells. We found that in Y79 and SO-RB50 cell lines, compared with mimic control+NC group, ECM1 protein level was highly expressed in mimic control+ECM1 group, and lowly expressed in mimic+NC group (Figure 6A-C, *P*<0.05). At the same time, ECM1 protein level in mimic+ECM1 group was lower than that in mimic control+ECM1 group but was higher than that in mimic+NC group (Figure 6A-C, *P*<0.05). ECM1 level was inhibited by miR-486-3p mimic in RB cells, and ECM1 vectors restored the ECM1 expression.

**Figure 6:** The role of miR-486-3p combined with ECM1 in RB cells was observed (**A**) Y79 was co-transfected with miR-486-3p mimic and ECM1 or their negative control (mimic control+NC group, mimic control+ECM1 group, mimic+NC group, mimic+ECM1 group), the ECM1 protein level was detected by Western blot. (**B**) SO-RB50 was co-transfected with miR-486-3p mimic and ECM1 or their negative control (mimic control+NC group, mimic control+ECM1 group, mimic+NC group, mimic+ECM1 group), the ECM1 protein level was detected by Western blot. (**C**) The miR-486-3p mimic decreased ECM1 level, while ECM1 reversed the effect of the miR-486-3p mimic. (**D**) Cell viability of Y79 and SO-RB50 was determined by CCK-8. (**E**) Apoptosis of Y79 and SO-RB50 was determined by flow cytometry. (**F**) In Y79 and SO-RB50, ECM1 inhibited apoptosis, and partially reversed the promoting effect of miR-486-3p on apoptosis. (**G**) Cloning ability of Y79 and SO-RB50 cells was determined by clone formation assay. (**H**) ECM1 increased cell cloning and partially reversed the inhibitory effect of miR-486-3p on cell cloning. *P<0.05 and **P<0.01 vs. mimic control+NC;^ #^*P*<0.05 and ^##^*P*<0.01 vs. mimic control+ECM1; ^^^*P*<0.05 and ^∧∧^*P*<0.01 vs. mimic+NC.

RETRACTED

### ECM1 reversed the effect of miR-486-3p on RB cells

The cell proliferation, apoptosis, migration and invasion of transformed Y79 and SO-RB50 were determined by CCK-8, clone formation assay, flow cytometry, scratch and transwell. Compared with mimic control + NC group, cell viability (Figure 6D), clones (Figure 6G,H), migration (Figure 7A,B) and invasion (Figure 7C,D) were up-regulated in mimic control+ECM1 groups and down-regulated in mimic+NC group (*P*<0.05). The cell viability (Figure 6D), clones (Figure 6G,H), migration (Figure 7A,B) and invasion (Figure 7C,D) in mimic+ECM1 group were higher than those in mimic+NC group and lower than those in mimic control+ECM1 group (*P*<0.05). In addition, the apoptosis in mimic+NC group was up-regulated as compared with mimic control+NC group, and the apoptosis in mimic+ECM1 group was higher than that in mimic control+ECM1 group but was lower than that in mimic+NC group (Figure 6E,F, *P*<0.05). ECM1 could promote cell proliferation, migration and invasion, and inhibit apoptosis, as well as reverse the effect of miR-486-3p on RB cells. The miR-486-3p may play a role in RB by regulating ECM1 expression.

**Figure 7:** The role of miR-486-3p combined with ECM1 in migration and invasion of RB cells was observed (**A**) Cell migration of Y79 and SO-RB50 was determined by scratch assay. (**B**) In Y79 and SO-RB50, cell migration was promoted by ECM1, and ECM1 reversed the inhibitory effect of miR-486-3p on cell migration. (**C**) In Y79 and SO-RB50, cell invasion was promoted by ECM1, and ECM1 reversed the inhibitory effect of miR-486-3p on cell invasion. (**D**) Cell invasion of Y79 and SO-RB50 was determined by transwell. *P<0.05 and **P<0.01 vs. mimic control+NC; ^##^*P*<0.01 vs. mimic control +ECM1; ^∧∧^*P*<0.01 vs. mimic+NC.

## Discussion

In the present study, we found that miR-486-3p level was down-regulated in RB tissues and cells, suggesting that miR-486-3p was involved in the development of RB. Venkatesan et al. [27] also found that the miR-486-3-p expression was down-regulated in RB samples. Then, *in vitro* experiments were conducted, and demonstrated that miR-486-3p overexpression inhibited the proliferation, migration and invasion, and promoted the apoptosis of RB. At the same time, the downstream target gene of miR-486-3p was analyzed and verified, and found ECM1 was the target gene of miR-486-3p and ECM1 expression was suppressed by overexpressed miR-486-3p. Finally, the role of miR-486-3p combined with target gene in RB cells was observed, and found that overexpression of ECM1 partially reversed the effect of miR-486-3p on RB cells. These results support the conclusion that miR-486-3p plays a crucial role in RB progression.

RETRACTED

Continuous proliferation of tumor cells is one of the basic biological characteristics of tumor progression [28]. In normal conditions, the cell proliferation and apoptosis are in a dynamic equilibrium state, and abnormal cell growth or death can lead to tumor or excessive tumor cells [29]. In addition, tumor metastasis is an important cause for poor prognosis of cancer patients, and important biological characteristics of tumor metastasis are cell migration and invasion [30]. Tumor cells can enter the microcirculation through the microvessels and lymphatic vessels, and invade into the surrounding tissues, resulting in tumor metastasis [31,32]. In this study, the role of miR-486-3p on the proliferation, migration and invasion of RB cells was investigated, and the result showed that overexpression of miR-486-3p could inhibit the cell proliferation, migration and invasion of RB cells. The results revealed that miR-486-3p may play an anticancer role in RB. In other studies, miR-486-3p has been reported to have an inhibitory effect on cancer, such as glioblastoma [33], oral cancer [24] and cervical cancer [25].

In addition, the occurrence of cancer is closely related to the abnormal apoptosis regulation mechanics, which may lead to the increase in the number of tumor cells [34,35]. Meanwhile, the occurrence of apoptosis is a complex process, which is strictly regulated by many genes, including pro-apoptotic genes and apoptotic suppressor genes [36]. Bax is the most widely studied pro-apoptotic protein, which can form heterodimer with Bcl-2 (an anti-apoptotic protein), thus acting as apoptotic activator [37]. Caspase-3 belongs to the apoptotic effector gene, and the activated caspase-3 will trigger a cascade reaction, leading to irreversible apoptosis [38]. In this study, it was found that miR-486-3p promoted the apoptosis of RB cells by down-regulating the Bcl-2 level, increasing the Bax level and activating caspase-3, and thereby inhibiting the malignant progression of RB.

RETRACTED

MiRNAs participate in a variety of physiological and pathological processes by regulating their multiple target genes [39]. It has been reported that miR-486-3p plays a critical role in proliferation and metastasis by repressing various oncogenes, including DDR1 [24] and BMP2 [40]. To further clarify the mechanism of miR-486-3p in RB, the target gene of miR-486-3p was identified. In the present paper, ECM1 was identified as the functional target of miR-486-3p in RB cells. ECM1 was as a ‘biological glue’ binding to components of the dermal–epidermal junction in the framework of normal skin [41]. ECM1 was first found in osteoblasts stromal cells, and high ECM1 levels were subsequently detected in bladder cancer [42], thyroid cancer [43] and other malignant tumors [44]. Chen et al. [45] showed that ECM1 was highly expressed in hepatocellular carcinoma specimens, and could promote the migration and invasion of HCC cells. In cervical cancer, miR-486-3p inhibited cell proliferation by targeting ECM1 [25]. We discovered that the overexpression of miR-486-3p significantly inhibited the ECM1 expression in RB cells, ECM1 could partially reverse the effects of miR-486-3p on RB cells, and promote cell proliferation, while inhibit apoptosis. The above results indicated that miR-486-3p may play a tumor suppressive role in RB through inhibiting the ECM1 expression.

In conclusion, miR-486-3p expression was decreased in RB tissues and participated in the development of RB. Moreover, miR-486-3p inhibited the cell proliferation, migration and invasion, and promoted apoptosis by inhibiting ECM1 expression, thus inhibiting the malignant progression of RB. The present study suggests that miR-486-3p may be a potential therapeutic target for clinical treatment of RB.

## Abbreviations

Bax: Bcl2-associated X
Bcl-2: B-cell lymphoma-2
BMP2: bone morphogenetic protein-2
C caspase-3: cleaved caspase-3
CCK-8: cell counting kit-8
DDR1: discoidin domain receptor-1
DRAM2: DNA-damage-regulated autophagy modulator protein
ECM1: extracellular matrix protein 1
FBS: fetal bovine serum
GAPDH: glyceraldehyde-3-phosphate dehydrogenas
HRP: horseradish peroxidase
miRNA: microRNA
OD: optical density
qRT-PCR: quantitative real-time polymerase chain reaction
RB: retinoblastoma
3′-UTR: 3′-untranslation region
